# Long noncoding RNA SNHG1 promotes TERT expression by sponging miR-18b-5p in breast cancer

**DOI:** 10.1186/s13578-021-00675-5

**Published:** 2021-08-31

**Authors:** Yujuan Kang, Lin Wan, Qin Wang, Yanling Yin, Jiena Liu, Lei Liu, Hao Wu, Lei Zhang, Xin Zhang, Shouping Xu, Da Pang

**Affiliations:** 1 Department of Breast Surgery, Harbin Medical University Cancer Hospital, Harbin, 150040 China; 2 Heilongjiang Academy of Medical Sciences, Harbin, China

**Keywords:** SNHG1, TERT, Breast cancer, Competing endogenous RNA, E2F1

## Abstract

**Background:**

Long noncoding RNA (lncRNA) small nucleolar RNA host gene 1 (SNHG1) plays a positive role in the progression of human malignant tumors. However, the molecular mechanism of SNHG1 remains elusive in breast cancer.

**Results:**

LncRNA SNHG1 was upregulated and had a positive relationship with poor prognosis according to bioinformatics analysis in pan-cancer including breast cancer. Silencing SNHG1 inhibited tumorigenesis in breast cancer both in vitro and in vivo. Mechanistically, SNHG1 functioned as a competing endogenous RNA (ceRNA) to promote TERT expression by sponging miR-18b-5p in breast cancer. miR-18b-5p acted as a tumor repressor in breast cancer. Moreover, the combination of SNHG1 knockdown and TERT inhibitor administration showed a synergistic inhibitory effect on breast cancer growth in vivo. Finally, E2F1 as a transcription factor, binding to SNHG1 promoter and enhanced SNHG1 transcription in breast cancer.

**Conclusions:**

Our results provide a comprehensive understanding of the oncogenic mechanism of lncRNA SNHG1 in breast cancer. Importantly, we identified a novel E2F1–SNHG1–miR-18b-5p–TERT axis, which may be a potential therapeutic target for breast cancer. Our results also provided a potential treatment for breast cancer when knockdown SNHG1 and TERT inhibitor administration simultaneously.

**Supplementary Information:**

The online version contains supplementary material available at 10.1186/s13578-021-00675-5.

## Background

Long noncoding RNAs (lncRNAs) are a large family of RNAs with limited protein-coding potential, length of over 200 nucleotides, and lack of a detectable open reading frame [1–5]. Importantly, lncRNA dysregulation has been observed in various cancers, and they reportedly participate in cancer cell growth, metastasis, and drug resistance [6, 7]. Moreover, lncRNAs are a novel class of potential biomarkers and therapeutic targets for cancer treatment [8]. In terms of regulatory mechanisms, when lncRNAs are located in the nucleus, they regulate gene expression by acting as epigenetic modulators [9, 10]; whereas, most lncRNAs in the cytoplasm harbor multiple binding sites for identical microRNAs (miRNAs), and are called competing endogenous RNAs (ceRNAs) [11]. miRNAs are a class of pervasive, conserved, small, noncoding RNAs that act as negative gene regulators to repress the expression of target genes [12]. ceRNAs can sequester miRNAs and protect the target mRNAs from being repressed [13, 14]. LncRNA small nucleolar RNA host gene 1 (SNHG1) is localized at 11q12.3 and shows upregulated expression in various cancers, including glioma and lung cancer [15–17]. In addition, SNHG1 reportedly serves as an oncogene in human cancers including breast cancer [18]. For instance, Cui et al. have shown that SNHG1 promotes the progression of pancreatic cancer via the Notch-1 signaling pathway [19]. Pei et al*.* has showed that interference SNHG1 inhibited the differentiation of Treg cells by promoting miR-448 expression and regulating IDO level, thereby impeding the immune escape of breast cancer [20]. Xiong et al*.* showed that SNHG1 promotes breast cancer progression by regulating of LMO4 [21]. Li et al. SNHG1 activates HOXA1 expression via sponging miR-193a-5p in breast cancer progression [22]. Zheng et al*.* SNHG1 contributes to proliferation and invasion by regulating miR-382 in breast cancer [23].

Telomeres are cellular nucleoprotein complexes that maintain chromosomal integrity and genome stability [24]. Telomeres are formed by hexameric repeats of a 5′-TTAGGG-3′ sequence ending in a 3′ single-stranded overhang, the G-strand overhang [25, 26] that protects the genomic DNA from the continued erosion of telomeres during cell division. Human telomerase is composed of two main core subunits: TERT, which constitutes the catalytic subunit and telomerase RNA component, which provides a template for telomerase elongation [27–29]. Human TERT protein levels are rate-limiting for telomerase activity and telomere length homeostasis [30]. A positive correlation between TERT mRNA expression and telomerase activity has been observed, thereby suggesting that telomerase is primarily regulated by TERT gene expression [28, 31, 32]. In approximately 90% of human tumors, telomerase is either upregulated or reactivated to maintain the telomeres during numerous rounds of cell divisions that are required for the emergence of malignant and metastatic diseases [33]. In cancer cells, TERT activity shows differential upregulation that is possibly due to several processes, such as transcriptional regulation, alternate RNA splicing, and post-translational modifications such as protein phosphorylation [30, 34]. Breast cancer is one of the leading mortal causes from cancer among women worldwide [35, 36]. Surgery, radiotherapy, chemotherapy and hormone therapy are still the main and common therapeutic approaches to treat breast cancer [37]. It was reported that the mRNA expression of TERT in breast cancer samples has a positive relationship with poor prognosis [38]. However, to date, no studies have determined the mechanism of the relationship between SNHG1 and TERT in breast cancer. Thus, in this study, we attempted to elucidate the oncogenic function of SNHG1 in breast cancer. To the best of our knowledge, this is the first study to report that a E2F1–SNHG1–miR-18b-5p–TERT axis is involved in breast cancer, and this axis may be a novel potential therapeutic target for the same. Moreover, the combination of SNHG1 knockdown and TERT inhibitor administration may be a potential treatment for breast cancer.

## Results

### Expression of SNHG1 was upregulated in cancerous tissues and positively related to poor prognosis

To determine the expression level of SNHG1 in human pan-cancer tissues, TCGA data was downloaded and analyzed. SNHG1 expression level was higher in thyroid carcinoma (THCA), stomach adenocarcinoma (STAD), sarcoma (SARC), rectum adenocarcinoma (READ), prostate adenocarcinoma (PRAD), pheochromocytoma and paraganglioma (PCPG), lung squamous cell carcinoma (LUSC), lung adenocarcinoma (LUAD), liver hepatocellular carcinoma (LIHC), kidney renal papillary cell carcinoma (KIRP), kidney renal clear cell carcinoma (KIRC), kidney chromophobe (KICH), head and neck squamous cell carcinoma (HNSC), esophageal carcinoma (ESCA), colon adenocarcinoma (COAD), cholangiocarcinoma (CHOL), cervical squamous cell carcinoma and endocervical adenocarcinoma (CESC), breast invasive carcinoma (BRCA) (Additional file 3: Table S1), bladder urothelial carcinoma (BLCA) than in normal tissues (Fig. 1a and Additional file 4: Table S2). Furthermore, the expression of SNHG1 was also more upregulated in pan-cancer tissues than in normal tissues (Fig. 1b). We also examined five pairs of breast cancer tissues and normal breast tissues to determine SNHG1 expression and observed that SNHG1 showed higher expression level in breast cancer tissues than in paired normal tissues (Fig. 1c and Additional file 5: Table S3). The PrognoScan database demonstrated that higher expression level of SNHG1 was associated with poor relapse-free survival (RFS) (Fig. 1d), and disease-specific survival (DSS) (Fig. 1e) in patients with breast cancer. In pan-cancer analysis, upregulated SNHG1 expression was also related to poor overall survival (OS) and DSS (Fig. 1f, g, Additional file 4: Table S2). Moreover, higher expression of SNHG1 also correlated with poor prognosis in UCEC, LIHC, PRAD, and adrenocortical carcinoma (ACC) (Additional file 1: Fig. S1a–k and Additional file 4: Table S2). We use the KM plotter (http://kmplot.com/analysis/) to evaluate the prognostic value of SNHG1 in different cancers [39]. Higher expression of SNHG1 was correlated with poor OS in LIHC, KIRC, SARC and UCEC (Additional file 1: Fig. S1l–o).

**Fig. 1:** Expression of SNHG1 was upregulated in cancerous tissues and positively related to poor prognosis. **a** The Cancer Genome Atlas results showed that the expression level of SNHG1 was higher in THCA, STAD, SARC, READ, PRAD, PCPG, LUSC, LUAD, LIHC, KIRP, KIRC, KICH, HNSC, ESCA, COAD, CHOL, CESC, BRCA, BLCA than in normal tissues. **b** Expression level of SNHG1 was also higher in pan-cancer tissues than in normal tissues. **c** Expression level of SNHG1 was higher in breast cancer tissues than in normal tissue (N = 5 per group). **d**, **e** PrognoScan results showed that higher SNHG1 expression level had a positive association with poor overall survival (OS), relapse-free survival (RFS), and disease-specific survival (DSS) in breast cancer. **f**, **g** Higher expression level of SNHG1 was related to poorer OS and DSS according to pan-cancer analysis. *P < 0.05; **P < 0.01; ***P < 0.001; *****P < 0.0001; *NS* no significance

### SNHG1 as an oncogene promoted tumorigenesis both in vitro and in vivo

Hs578T, MDA-MB-468, and MDA-MB-231 are breast cancer cell lines that have higher SNHG1 expression level than MCF10A cells (Fig. 2a); consequently, they were chosen for subsequent experiments. SNHG1 was knocked down by transfection with siSNHG1, and the transfection efficiency of siSNHG1 was evaluated using reverse transcription-polymerase chain reaction (RT-PCR) (Fig. 2b). Further, cell counting kit-8 (CCK-8), colony formation, wound healing, and Transwell invasion assays were performed to identify the function of SNHG1 in breast cancer. We observed that silencing of SNHG1 inhibited tumor cell proliferation, colony formation and suppressed tumor cell migration and invasion (Fig. 2c–f).

**Fig. 2:** SNHG1 acts an oncogene promoted tumorigenesis both in vitro and in vivo. **a** Expression of SNHG1 in MCF10A, Hs578T, MDA-MB-231, and MDA-MB-468 cell lines. **b** Transfection efficacy of siSNHG1 in MDA-MB-468, Hs578T, and MDA-MB-231 cells. **c** CCK-8 showed that silencing SNHG1 inhibited tumor cell proliferation. **d** Colony formation assay showed that silencing SNHG1 inhibited tumor cell clone formation. **e** Wound healing assay proved that silencing SNHG1 suppressed tumor cell migration. **f** Transwell invasion assay showed that knockdown of SNHG1 inhibited the invasion ability of tumor cells. **g** Knockdown efficacy of lentiviral targeting of snhg1. **h** CCK-8 showed that silencing of snhg1 suppressed 4T1 proliferation. **i** Tumor growth curve of mice shows that sh-snhg1#3 group had slower growth than that in the scramble group. **j** Tumor weight in the sh-snhg1#3 group was lower than that in the scramble group. **k** The tumorigenesis and tumor tissue of each group of Balb/C mice (N = 6 per group) are shown. **l** The survival of scramble and sh-snhg1#3 mice (N = 6 per group). Data are presented as the mean value from three independent experiments ± S.D. *P < 0.05; **P < 0.01; ***P < 0.001; *****P < 0.0001; *NS* no significance

Subsequently, we evaluated the functions of SNHG1 in vivo. Lentivirus was synthesized to construct a 4T1 stable knockdown of snhg1 (sh-snhg1). Knockdown efficiency was determined using RT-PCR, and we observed that the virus could knockdown snhg1 in 4T1, as expected (Fig. 2g). The CCK-8 assay showed that the sh-snhg1 group had poorer proliferation ability than the scramble group (Fig. 2h). Further, 4T1 scramble and 4T1 sh-snhg1#3 cells were subcutaneously injected into Balb/C female mice. As expected, the mice from the sh-snhg1#3 group had smaller tumors than those from the scramble group (Fig. 2i), thereby suggesting that SNHG1 acted as an oncogene in vivo as well. Moreover, the median tumor weight in the sh-snhg1#3 group was lower than that in the control group (Fig. 2j). The tumorigenesis and tumor tissue of each group of Balb/C mice are shown as Fig. 2k. Furthermore, we pay attention to the relationship between SNHG1 expression and survival. The animal experiment results showed that sh-snhg1#3 group mice have a longer survival compared with scramble group (N = 8) (Fig. 2l). Thus, the abovementioned results showed that SNHG1 acted as an oncogene in breast cancer both in vitro and in vivo.

### SNHG1 boosted TERT expression

Then, TCGA data was downloaded to evaluate the correlation between SNHG1 and TERT in pan-cancer and breast cancer. The results showed that TERT is positively correlated with SNHG1 in pan-caner scope (R = 0.2945) and breast cancer scope (R = 0.3685) (Fig. 3a, b and Additional file 6: Table S4). In addition, the Gene Expression Profiling Interactive Analysis (GEPIA) was used to verify this relationship, and the results showed that TERT was positively correlated with SNHG1 (Fig. 3c).

**Fig. 3:** SNHG1 boosted TERT expression. TCGA data showed that TERT is positively correlated with SNHG1 in pan-caner (N = 9725) (**a**) and in breast cancer (N = 1097) (**b**). **c** GEPIA showed that TERT expression level was higher in breast cancer tissues than in normal tissues. **d**, **e** We identified that TERT gene was upregulated expressed between high SNHG1 group and low SNHG1 group with FDR = 4.45785008467688e−19, FC = 0.418132443350429 in breast cancer. **f** GEPIA showed that the expression of TERT a higher level in breast cancer tissue than that in normal tissue. **g** TERT presents a higher expression level in breast cancer cell lines than in MCF10A cell. **h** TERT showed higher expression level in breast cancer tissues than in paired normal tissues in our own cohort (N = 4 per group). **i** Transfection efficacy of siSNHG1. **j** Knockdown of SNHG1 downregulated TERT mRNA expression in Hs578T and MDA-MB-468 cells. Knockdown of SNHG1 also downregulated TERT protein expression in MDA-MB-468 and Hs578T cells (**k**). **l** The transfection efficiency of SNHG1 plasmid. **m**, **n** The expression of TERT RNA and protein upregulated after SNHG1 overexpression. **o** TERT protein had a higher expression level in the scramble group than in the sh-snhg1#3 group. **p**–**r** The tumorigenesis, tumor tissue, tumor growth and tumor weight of 4T1 cells in each group of Balb/C mice (N = 6 per group) are shown. Data are presented as the mean value from three independent experiments ± S.D. *P < 0.05; **P < 0.01; ***P < 0.001; *****P < 0.0001; *NS* no significance

Moreover, according to SNHG1 gene expression level, BRCA cancer tissue samples were divided into two groups: SNHG1 high expression group SNHG1 low expression group. We identified a total of 595 differential expressed genes (FDR < 0.01, fold change > 1.2), among which 456 genes were upregulated and 139 genes were downregulated (Fig. 3d, e and Additional file 7: Table S5). TERT gene was upregulated expressed between high group and low group with FDR = 4.45785008467688e−19, FC = 0.418132443350429. As TERT was a certain target gene of SNHG1 in breast cancer, we select it as the SNHG1 downstream gene.

The GEPIA database showed that TERT expression level was considerably higher in breast cancer tissues than in normal tissues (Fig. 3f). Just as Fig. 3g showed, TERT presents a higher expression level in breast cancer cell lines than in MCF10A cell. We then examined four pairs of breast cancer tissues and normal breast tissues to determine TERT expression and observed that TERT showed higher expression level in breast cancer tissues than in paired normal tissues (Fig. 3h and Additional file 5: Table S3). Moreover, CCK-8, colony formation and wound healing assays were performed to identify the function of TERT in breast cancer. We observed that silencing of TERT inhibited tumor cell proliferation and colony formation and tumor cell migration ability (Additional file 2: Fig. S2a–c).

SiSNHG1 was transfected into MDA-MB-468 and Hs578T, and RT-PCR was used to examine the transfection efficiency of siSNHG1 (Fig. 3i). Consequently, we observed that knockdown of SNHG1 downregulated the expression of TERT at both RNA (Fig. 3j) and protein levels (Fig. 3k) in MDA-MB-468 and Hs578T cells in comparison to their levels in corresponding control groups. To validate the regulatory axis through a contrasting approach, we also transfected SNHG1 overexpression plasmid to MDA-MB-468 and Hs578T. RT-PCR was used to confirm the transfection efficiency (Fig. 3l). The expression of TERT in RNA and protein level is upregulated in SNHG1 overexpression group compared to control group (Fig. 3m, n). Furthermore, for the in vivo experiment, we extracted protein and RNA from mouse tumors and observed that the expression level of TERT in mouse tumors was lower in the sh-snhg1#3 group than in the control group (Fig. 3o).

Thus, SNHG1 promoted TERT expression in breast cancer. Next, we wondered whether targeting SNHG1 and TERT could produce a synergistic inhibitory effect. BIBR1532 is a nonnucleotidic small molecule compound that selectively inhibits telomerase activity by competitively binding to the active site of hTERT [40]. As we expected, the combination of knocking down snhg1#3 and administering the BIBR1532 (TERT inhibitor) prohibited tumor growth more powerfully than either approach alone (Fig. 3p, q). The median weight in the combination group was lower than that in the snhg1 knockdown group or control group (Fig. 3r).

### miR-18b-5p acted as a tumor suppressor in breast cancer

We further explored the mechanism by which SNHG1 promoted the expression of TERT in breast cancer. First, LncLocator was used to predict the subcellular localization of SNHG1, and the results showed that SNHG1 was mainly localized in the cytoplasm (Fig. 4a). Then, a cytoplasmic-nuclear RNA fractionation kit was used to confirm the forward prediction results in HEK293T, MDA-MB-468, and Hs578T cells (Fig. 4b). Both methods implied that SNHG1 was mainly localized in the cytoplasm. Therefore, we hypothesized that cytoplasmic SNHG1 might regulate TERT mRNA by acting as a ceRNA of miRNAs. To confirm this hypothesis, we used miRbase, TargetScan, and starBase databases to predict the possible miRNAs that could interact with both SNHG1 and TERT, simultaneously (Additional file 8: Table S6). The intersection of miRNAs acquired from these databases revealed 15 overlapping miRNAs (Fig. 4c). RT-PCR was used to determine the upregulated miRNAs after silencing SNHG1 in MDA-MB-468 and Hs578T cells (Fig. 4d, e). Finally, miR-18b-5p and miR-383-5p were chosen for subsequent experiments. However, when miR-383-5p mimics were transfected into Hs578T cells, the expression of TERT was upregulated (Fig. 4f). Thus, miR-18b-5p was the only candidate for subsequent experiments. Moreover, after SNHG1 overexpression, the expression of miR-18b-5p also downregulated when compared with control group in MDA-MB-468 and Hs578T (Fig. 4g). To explore the functions of miR-18b-5p in breast cancer, we performed CCK-8, colony formation, wound healing, and Transwell invasion assays by transfecting Hs578T, MDA-MB-468, and MDA-MB-231 cells with miR-18b-5p mimics. The transfection efficiency of miR-18b-5p mimics was verified by RT-PCR (Fig. 4h), and cell proliferation and colony formation were attenuated on transfecting miR-18b-5p mimics (Fig. 4i, j). Further, wound healing and Transwell invasion assays showed that overexpression of miR-18b-5p could inhibit tumor cell migration and invasion (Fig. 4k, l). Thus, the abovementioned experiments indicated that miR-18b-5p may act as a tumor suppressor in breast cancer.

**Fig. 4:** miR-18b-5p acted as a tumor suppressor in breast cancer. **a** LncLocator predicted the subcellular localization of SNHG1. **b** Subcellular RNA fraction confirmed that SNHG1 was mainly located in the cytoplasm in HEK293T, MDA-MB-468, and Hs578T cells. **c** The intersection of TargetScan and StarBase predicted miRNAs. **d**, **e** The upregulated miRNAs after silencing of SNHG1 in MDA-MB-468 and Hs578T cells. **f** Expression of TERT after transfecting miR-383-5p mimics in Hs578T cells. **g** The expression of miR-18b-5p was downregulated after SNHG1 overexpression. **h** Transfection efficiency of miR-18b-5p mimics in Hs578T, MDA-MB-468, and MDA-MB-231 cells. **i** Colony counting kit-8 proved that miR-18b-5p inhibited cell proliferation. **j**–**l** Colony formation assay, wound healing assay and Transwell invasion assay showed that miR-18b-5p inhibited breast cancer cell colony formation, migration and invasion. Data are presented as the mean value from three independent experiments ± S.D. *P < 0.05; **P < 0.01; ***P < 0.001; *****P < 0.0001; *NS* no significance

### SNHG1 acted as a ceRNA to enhance TERT expression by sponging miR-18b-5p

We further explored the regulatory mechanism of SNHG1, miR-18b-5p, and TERT in breast cancer. RT-PCR was used to evaluate the transfection efficiency of miR-18b-5p mimics (Fig. 5a). TERT RNA level was downregulated after transfecting miR-18b-5p mimics (Fig. 5b); whereas, the TERT RNA level was upregulated after transfecting miR-18b-5p inhibitor (Fig. 5d). Accordingly, TERT protein level was downregulated after transfecting miR-18b-5p mimics (Fig. 5c), and upregulated after transfecting miR-18b-5p inhibitor (Fig. 5e). Furthermore, overexpression of miR-18b-5p inhibited SNHG1 expression; however, downregulation of miR-18b-5p promoted SNHG1 expression in MDA-MB-468 and Hs578T cells (Fig. 5f, g). Moreover, silencing SNHG1 and inhibiting miR-18b-5p weakened the downregulation of TERT protein level in MDA-MB-468 and Hs578T cells (Fig. 5h). Finally, the dual-luciferase reporter assay was used to demonstrate the binding relationship between SNHG1, miR-18b-5p, and TERT. As expected, wild-type 3′-untranslated region of TERT was regulated by miR-18b-5p, and this effect could be neutralized by mutating the binding sites in the luciferase reporter (Fig. 5i). Additionally, we obtained similar results for the regulation of SNHG1 (Fig. 5j). SNHG1 function was partially mediated by inhibiting miR-18b-5p in breast cancer cells. We transfected siSNHG1 and miR-18b-5p inhibitor into breast cancer cells and observed that siSNHG1-mediated restraint in cell proliferation and invasion abilities could be partially rescued by co-transfection of miR-18b-5p inhibitor in Hs578T and MDA-MB-468 cells (Fig. 5k, l). In addition, the expression of miR-18b-5p was more upregulated in in Balb/C mice with snhg1 knockdown than in the scramble group (N = 5) (Fig. 5m), which was consistent with our previous conclusion. Thus, SNHG1 upregulated the expression of TERT via a ceRNA mechanism by sponging miR-18b-5p in breast cancer.

**Fig. 5:** SNHG1 acted as a ceRNA to enhance TERT expression by sponging miR-18b-5p. **a** Transfection efficacy of miR-18b-5p mimics in MDA-MB-468 and Hs578T cells. **b**, **c** Overexpression of miR-18b-5p downregulated TERT mRNA and protein expression. **d**, **e** miR-18b-5p inhibitor upregulated TERT mRNA and protein expression. **f**, **g** Overexpression of miR-18b-5p inhibited SNHG1 expression; however, downregulated miR-18b-5p promoted SNHG1 expression. **h** Silencing SNHG1 and inhibiting miR-18b-5p weakened the downregulation of TERT at the protein level in MDA-MB-468 and Hs578T cells. **i**, **j** A luciferase reporter assay was used to assess the interactions between miR-18b-5p and its binding sites or mutated binding sites in the 3′ UTRs of TERT and SNHG1 in HEK293T cells. **k**, **l** siSNHG1-mediated restraint of cell proliferation and invasion abilities was partially rescued by co-transfection of miR-18b-5p inhibitor in Hs578T and MDA-MB-468 cells. **m** miR-18b-5p expression in Balb/C mice with snhg1 knockdown. Data are presented as the mean value from three independent experiments ± S.D. *P < 0.05; **P < 0.01; ***P < 0.001; *****P < 0.0001; *NS* no significance

### E2F1 promoted SNHG1 transcription

We further focused on elucidating the upstream transcription regulation mechanism of SNHG1. First, PROMO database was used to predict potential transcription factors (TFs) that could bind to the SNHG1 promoter (Additional file 9: Table S7). We focused on E2F1, a prominent TF that mediates transcriptional activation in a variety of tumors. TCGA data was downloaded to evaluate the correlation between E2F1 and SNHG1 in pan-cancer and breast cancer. The results showed that E2F1 is positively correlated with SNHG1 in pan-caner (R = 0.4129) and breast cancer (R = 0.3521) (Fig. 6a and Additional file 10: Table S8). To verify this prediction, we transfected MDA-MB-468, Hs578T, and HEK293T cells with an siRNA to silence E2F1. Knockdown efficiency was examined by RT-PCR (Fig. 6b) and western blotting analysis (Fig. 6c). RT-PCR showed that the expression level of SNHG1 (Fig. 6d) and TERT (Fig. 6e) in the siE2F1 group was lower than that in the control group. Moreover, the expression of miR-18b-5p is increased after silencing E2F1 (Fig. 6f). Further, the JASPAR database was used to predict the potential binding site between E2F1 and SNHG1 promotor (Fig. 6g, h, Additional file 11: Table S9). Finally, chromatin immunoprecipitation-PCR assay indicated that in comparison with the Mock group, E2F1 was enriched at the SNHG1 promoter in Hs578T and HEK293T cells (Fig. 6i). Overall, we found a regulatory axis, E2F1–SNHG1–miR-18b-5p–TERT, play a vital role in breast cancer. Then, we found that when silencing TERT in MDA-MB-468 and Hs578T, the expression of SNHG1 decreased and the expression of miR-18b-5p upregulated. There may be a circle regulation mechanism between SNHG1 and TERT in breast cancer which deserved to excavate in the future (Fig. 6j, k). A schematic illustration of this study is shown in Fig. 6l.

**Fig. 6:** E2F1 promoted SNHG1 transcription. **a** TCGA data showed that E2F1 is positively correlated with SNHG1 in pan-caner and in breast cancer. Knockdown efficacy of siE2F1 at mRNA (**b**) and protein (**c**) levels in MDA-MB-468, Hs578T, and HEK293T cells. **d** Knockdown of E2F1 downregulated SNHG1 expression. **e** Knockdown of E2F1 downregulated TERT mRNA expression. **f** Knockdown of E2F1 upregulated miR-18b-5p expression. **g** JASPAR predicted that E2F1 could bind with the promoter of SNHG1. **h** Schematic representation of the predicted E2F1 binding sites within the promoter of SNHG1. **i** Chromatin immunoprecipitation assay showed the binding of E2F1 and SNHG1 promoter region in Hs578T and HEK293T cells. **j**, **k** Silencing TERT could downregulated the expression of SNHG1 and upregulated the expression of miR-18b-5p. **l** Working model of the study. Data are presented as the mean value from three independent experiments ± S.D. *P < 0.05; **P < 0.01; ***P < 0.001; *****P < 0.0001; *NS* no significance

## Discussion

Numerous studies have highlighted the functions of these regulatory lncRNAs in many biological processes, such as cancer development, stem cell differentiation, and chemotherapy resistance [41]. For instance, lncHOST2 act as a sponge of let-7b, thus increasing STAT3 expression and leading to breast cancer tumorigenesis [42]. SNHG1 promotes tumor growth by regulating the transcription of both local and distal genes [43]. TERT boosts epithelial-mesenchymal transformation and stemness, thereby indicating an important role in cancer progression [44]. This study revealed that SNHG1 was an oncogene that promoted the expression of TERT in breast cancer.

When lncRNAs are in the cytoplasm, they participate in modulating mRNA stability, regulating mRNA translation, serving as ceRNAs, and functioning as precursors of miRNAs [45]. Here, subcellular fractionation confirmed that SNHG1 was mainly located in the cytoplasm in breast cancer cell lines implying that SNHG1 acted as a ceRNA to enhance TERT expression by sponging miR-18b-5p in breast cancer.

To further explore the tumorigenesis mechanism of SNHG1 in breast cancer, we explored the upstream regulation of SNHG1. Notably, we observed that E2F1 could bind to the SNHG1 promoter and enhance its transcription in breast cancer. To summarize, this study uncovered a novel mechanistic axis, E2F1–SNHG1–miR-18b-5p–TERT, in breast cancer tumorigenesis, and this axis may be a potential therapeutic target for breast cancer. In addition, the combination of SNHG1 knockdown and TERT inhibitor administration showed a synergistic inhibitory effect on breast cancer growth which may provide a potential therapy for clinical therapy for breast cancer in near future. However, our study also has some limitations. Firstly, TERT might only be one of the many targets of miR-18b-5p and other targets gene should also be studied in future. Secondly, we have not studied the regulatory mechanism of SNHG1 which located in nucleus, and we will continue this study in near future. Thirdly, although SNHG1 was associated with shortened patients’ survival, it remains unclear if it can predict prognosis independent of other clinicopathological parameters, including age, sex and TNM staging.

## Conclusions

Our results identified a novel E2F1–SNHG1–miR-18b-5p–TERT axis, which may be a potential therapeutic target for breast cancer.

## Methods

### Public data access and analysis

Genome-wide SNHG1 expression profile and clinical pathology information for human cancers were downloaded from TCGA database (https://tcga-data.nci.nih.gov/). The transcript SNHG1 was normalized by log_2_ transformation. The expression of SNHG1 was dichotomized using a study-specific median expression as the cutoff to define “high value” at or above the median versus “low value” below the median. The detailed clinical pathological information including ID number, TNM stage of breast cancer patient from TCGA is shown in Additional file 3: Table S1. GEPIA database (http://gepia.cancer-pku.cn/) and TCGA database were used to predict the correlations between SNHG1 and TERT; E2F1 and SNHG1 in pan-cancer and breast cancer. Correlations between genes were assessed by Pearson correlation coefficients. Prognoscan (http://dna00.bio.kyutech.ac.jp/PrognoScan/index.html) [46] and KM plotter (http://kmplot.com/analysis/) were used to examine the survival of breast cancer patients according to differential SNHG1 expression level. The expression profile of coding gene in breast cancer was extracted from TCGA BRCA expression profile (Additional file 7: Table S5). According to SNHG1 expression level, breast cancer tissue samples were divided into two groups. SNHG1 high expression group was found to be more than or equal to the median value of SNHG1, while SNHG1 low expression group was found to be less than the median value. Differentially expressed gene (DEG) was identified by edgeR between SNHG1 high expression and low expression group, of which FDR < 0.01, FC > 1.2.

### Cell culture

MDA-MB-468, Hs578T, HEK293T, MDA-MB-231 and 4T1 cell lines were obtained from the Chinese Academy of Sciences Cell Bank. MDA-MB-468, Hs578T, HEK293T and 4T1 were cultured with DMEM medium (Gibco, Waltham, MA) and 10% fetal bovine serum (FBS; Gibco), 100 μ/mL penicillin and grown at 37 °C with 5% CO_2_ (Thermo). MDA-MB-231 was cultured with L15 (Gibco, Waltham, MA) medium and 10% FBS, 100 μ/mL penicillin and grown at 37 °C with air incubator (Thermo).

### Patients and tissue specimens

Breast cancer tissues and paired normal tissues were obtained from Harbin Medical University Cancer Center (HMUCC). None of the patients received adjuvant chemotherapy, immunotherapy, or radiotherapy before surgery, and patients with recurrent tumors, metastatic disease, bilateral tumors, or other previous tumors were excluded. For RNA extraction, fresh tissue from individuals with breast cancer and normal controls was collected and stored at − 80 °C immediately resection. The expression level of SNHG1 and TERT were measured by RT-qPCR. This study was approved by the Ethics Committees of Harbin Medical University. Written informed consent was obtained from all subjects who participated in this study.

### RNA extraction and RT-PCR

Total RNA samples from cells samples were isolated using Trizol reagent (Invitrogen, USA) according to manufacturer’s protocols. Total RNA (0.5 μg) was then reverse transcribed using Transcriptor First Strand cDNA Synthesis Kit (Roche, USA) to obtain cDNA. The SYBR Green PCR Master Mix Kit (Applied Biosystems, USA) was used to quantify the RNA levels using SYBR Green PCR Master Mix Kit, and the results were normalized against GAPDH and U6 expression levels using the 2^–ΔΔCT^ method. The RT-qPCR was performed on ABI StepOne Real-time PCR System (Applied Biosystems, USA). The primer sequences are as follows: SNHG1-F: 5′-AACTTCCCATAACTCCACTTC-3′; SNHG1-R: 5′-ACAACCAACACAGCAACAC-3′; TERT-F: 5′-CTGTACTTTGTCAAGGTGGATGTGA-3′; TERT-R: 5′-ACGTGTTCTGGGGTTTGATGATG-3′; Hsa-miR-18b-5p-F: 5′-CGGGCTAAGGTGCATCTAGTGC-3′; Hsa-miR-18b-5p-R: 5′-ATCCAGTGCAGGGTCCGAGG-3′; Hsa-miR-18b-5p-RT: 5′-GTCGTATCCAGTGCAGGGTCCGAGGTCCGAGGTATTCGCACTGGATACGACCTAACA-3′; Hsa-U6-F: 5′-GCTTCGGCAGCACATATACTAAAAT-3′; Hsa-U6-R: 5′-CGCTTCACGAATTTGCGTGTCAT-3′; Hsa-U6-RT: 5′-CGCTTCACGAATTTGCGTGTCAT-3′;

Hsa-miR-18a-5p-F: 5′-GCGGGCTAAGGTGCATCTAGTGC-3′; Hsa-miR-18a-5p-R: 5′-ATCCAGTGCAGGGTCCGAGG-3′; Hsa-miR-18a-5p-RT: 5′-GTCGTATCCAGTGCAGGGTCCGAGGTATTCGCACTGGATACGACCTATCT-3′; Hsa-miR-376a-3p-F: 5′-CGGGCCGGATCATAGAGGAAAAT-3′; Hsa-miR-376a-3p-R: 5′-ATCCAGTGCAGGGTCCGAGG-3′; Hsa-miR-376a-3p-RT: 5′-GTCGTATCCAGTGCAGGGTCCGAGGTATTCGCACTGGATACGACACGTGG-3′; Hsa-383-5p-F: 5′-GCGGGCAGATCAGAAGGTGATT-3′; Hsa-383-5p-R: 5′-ATCCAGTGCAGGGTCCGAGG-3′; Hsa-383-5p-RT: 5′-GTCGTATCCAGTGCAGGGTCCGAGGTATTCGCACTGGATACGACAGCCAC-3′; GAPDH-F: 5′-CATGTTCGTCATGGGTGTGAA-3′; GAPDH-R: 5′-GGCATGGACTGTGGTCATGAG-3′; E2F1-F: 5′-ACGTGACGTGTCAGGACCT-3′; E2F1-R: 5′-GATCGGGCCTTGTTTGCTCTT-3′; Mus-TERT-F: 5′-TCTACCGCACTTTGGTTGCC-3′; Mus-TERT-R: 5′-CAGCACGTTTCTCTCGTTGC-3′.

### Transfection of small interfering RNAs, miRNA mimics/inhibitors and plasmid

LncRNA SNHG1 short interfering RNA (siRNAs), Hsa-miR-18b-5p mimics and Hsa-miR-18b-5p inhibitor were synthesized by Ribo Co., Ltd. (Guangdong, China). SNHG1 plasmid (pcDNA3.1-SNHG1) was constructed by Shanghai GeneChem, Co. for SNHG1 overexpression. Cells were seeded in 6-well plate, when the cells grow 70–80% confluence for miRNA (100 nmol), siRNA (100 nmol), inhibitor (50 nmol) and SNHG1 overexpression plasmid (2000 ng) transfection. Cells were transfected using jetPRIME (Polyplus transfection). The sequences are as follows: si-control sense: UUCUCCGAACGUGUCACGUTT; si-SNHG1#1 sense: GGUUUGCUGUGUAUCACAUTT; si-SNHG1#2 sense: GACCUAGCUUGUUGCCAAUTT; si-E2F1#1 sense: GAGACCTCTTCGACTGTGA; si-E2F1#2 sense: CTATGAGACCTCACTGAAT; si-E2F1#3: GGGAGAAGTCACGCTATGA; si-TERT#1 sense: GAGCCAGTCTCACCTTCAA; si-TERT#2 sense: GGAGCAAGTTGCAAAGCAT; si-TERT#3 sense: GAGTGACCGTGGTTTCTGT. Scrambled negative control mimics/inhibitor and microRNA (miR) 18b-5p-, miR-383-5p were purchased from Invitrogen (Invitrogen, CA, USA) and had the following sequences: Hsa-miR-18b-5p mimics sense: UAAGGUGCAUCUAGUGCAGUUAG antisense: AACUGCACUAGAUGCACCUUAUU; Hsa-miR-18b-5p inhibitor sense: CUAACUGCACUAGAUGCACCUUA; Hsa-miR-383-5p mimics sense: AGAUCAGAAGGUGAUUGUGGCU antisense: CCACAAUCACCUUCUGAUCUUU; has-18b-5p inhibitor sense: CUAACUGCACUAGAUGCACCUUA.

### Lentiviral transfection

The full-length RNAi sequences and antisense were amplified by PCR and cloned into Lentiviral particles had puromycin selection and were constructed and packaged by Shanghai GeneChem, Co., Ltd. For lentiviral transfection, moderate lentiviruses were used to infect 4T1 cells in a 6-well plate with 4–6 µg/mL polybrene (#107689, Sigma). The infected cells were then subjected to selection with 1 µg/mL puromycin (#540411, Calbiochem, USA) cultured for several days. The stable knockdown of snhg1 was examined by RT-PCR. The sequence of lentivirus as follows: sh-snhg1#1: CTGGTGACAAATCTCAGGCAT; sh-snhg1#2: GTGGTTCATCTCAAAGCCCTT; sh-snhg1#3: AAGGATAGGAACAGAAATCAT.

### Cell viability assay

The viability of treated cells was estimated by a Cell Counting Kit-8 (CCK-8; Dojindo Laboratories, Kumamoto, Japan) assay according to the manufacturer’ instructions and as previous described [47]. Briefly, cells were plated at a density of 5 × 10^3^ cells/well with 100 μL of DMEM + 10% FBS in 96-well microtiter plates. 10 μL CCK-8 solution was added to each well which including 100 μL DMEM medium, and then the plate was incubated at 37 °C for 60 min. Next, the absorbance of each well was measured by a microplate reader at a wavelength of 450 nm. Medium containing 10% CCK-8 served as a control.

### Colony formation assay

1 × 10^3^ cells were seeded in 6-well plate and cultured in medium containing 10% FBS for 14 days.

Discard the culture medium, PBS wash the 6-well plate three times. Colonies were fixed with methanol for 40 min, then 500 μL of 5% crystal violet (Sigma-Aldrich, St. Louis, MO, USA) were added to each well for 30 min. After staining, colonies were gently washed and counted.

### Wound healing assay

Cells were seeded in 6-well plate, transfected with siRNAs or miRNA mimics according to previous method. When cell confluence reached 100%, 10 μL pipette was used to scratch on the bottom of the 6-well plate. The scratched cells were washed away. Then taking photos in 0 h, 24 h, 48 h.

### Transwell invasion assay

Transwell invasion assay was performed using a Transwell plate (Corning, New York, USA) was coated with Matrigel (Sigma-Aldrich, USA). 5 × 10^4^ cells in serum-free medium were suspended in upper chamber with Matrigel. Medium containing 20% FBS (Seratech, PAN) was added to the bottom chamber. After incubating at 37 °C for 48 h. Then discard the culture medium, cells that invaded to the lower side of the Transwell were fixed with methanol, stained with 0.5% crystal violet and imaged under a microscope. Image J was used to count the number of cells.

### Animal experiment

Animal experiments were approved by the Medical Experimental Animal Care Commission of Harbin Medical University. 4–5 weeks old female Balb/C mice were purchased from Animal Center of the Second Affiliated Harbin Medical University. 4T1 cells stably expressing sh-scramble and sh-snhg1#3 were resuspended with DMEM medium. Then 100 μL of serum-free medium containing 5 × 10^4^ cells were injected into the right mammary fat pad. The tumor volume was measured with a caliper every 2 days beginning on day 6 days after cell implantation. BIBR1532 was administrated intraperitoneally (i.p.) at a dose of 1.5 mg/kg for 2 weeks. The tumor volume was calculated using the formula tumor volume = 1/2 (length × width^2^). Then the mice were euthanized, the weight of tumors in mouse were measured. Then, half of the tumors was extracted protein and the other half was extracted RNA.

### Western blot assay

Cells were lysed with lysis buffer which containing 150 mmol/L NaCl, 1% Triton X-100, 5 mmol/L EDTA, 5000 U/mL aprotinin, 20 mg/mL leupeptin, 1 mmol/L phenyl-methylsulfonyl fluoride, 2 mmol/L sodium orthovanadate, 50 mmol/L NaF, 5% glycerol, 10 mmol/L Tris–HCl (pH 7.4), and 2% SDS. Then ultrasonic crusher was used to broken cell nucleus. After centrifugation at 13,500×*g* for 30 min, supernatant was collected. Next, protein concentrations were tested by BCA protein assay kit (#p0010; Beyotime, Shanghai, China). Then these proteins were separated by SDS-PAGE, followed by electroblotting onto a nitrocellulose membrane, which was blocked with 5% nonfat milk in 0.1% Tween 20-TBS overnight at 4 °C. The membrane was incubated with primary antibody against TERT (#sc-377511; Santa cruz biotechnology), E2F1 antibody (#3742; Cell Signaling Technology) and β-actin (#sc-377511; Santa cruz biotechnology). After washing with Tween 20/TBS (TBST), the membrane was incubated with horseradish peroxidase-conjugated secondary antibodies for 1 h in room temperature. After washing with Tween 20/PBS (PBST), protein bands on the membrane were visualized by an enhanced chemiluminescence Western blotting detection system (Western Lightning; Perkin-Elmer, Norwalk, CT).

### Dual-luciferase reporter gene assay

We cloned the full length of the 3′ untranslated regions (UTRs) of human SNHG1 and TERT to generate reporter vectors with miRNA binding sites. The full length of 3′ UTRs of human SNHG1 and TERT were amplified by PCR and cloned into psi-CHECK-2 luciferase expression vector that contained Not1-Xhol sites. HEK293T cells were chosen to perform this assay. When 293 T reached 40–50% confluence, JetPRIME was used to transfect HEK293T with 20 μmol/L Hsa-miR-18b-5p mimics or negative control mimics and 0.5 mg of plasmid. The luciferase activities were measured 48 h after transfection using a dual-luciferase reporter assay kit (#E1910, Promega, USA) and a luminometer (GloMax 20/20, Promega, USA).

### Cytoplasmic-nuclear RNA fractionation

Cytoplasmic and nuclear RNA extraction were separated using the cytoplasmic and nuclear RNA purification kit (#21000, NORGEN) as directed by the manufacturer. We harvested 3 × 10^6^ cells (HEK293T, MDA-MB-468, and Hs578T), washed them with ice-cold PBS, and then resuspended these cells in the ice-cold cytoplasmic Lysis Buffer J for 5 min on ice. Then lysates were centrifuged at 13,500×*g* for 10 min at 4 °C. The supernatant was collected as the cytoplasmic fraction, the remaining lysates was collected as the nuclear fraction. Finally, cytoplasm RNA and nucleus RNA were successfully separated. Then, the expression levels of GAPDH, U1 and SNHG1 in cytoplasm or nuclear were detected by RT-PCR.

### Chromatin immunoprecipitation (ChIP)

Chromatin immunoprecipitation (ChIP) assays were performed using the ChIP Assay Kit (#p2078; Beyotime, Shanghai, China) according to the manufacturer’s protocol. 2 × 10^7^ cells were crosslinked with 1% formaldehyde, and this reaction was terminated after 20 min by the addition of glycine at a final concentration of 0.125 M. DNA was immunoprecipitated from sonicated cell lysates using an E2F1 antibody; IgG (BD Biosciences, San Diego, CA, USA) served as the negative control. Protein A/G Plus-agarose was purchase from Santa cruz biotechnology (#sc-2003). R Nase A as Proteinase K treatment, immunoprecipitated DNA was extracted by DNA purification kit (Beyotime, Shanghai, China). The immunoprecipitated DNA was subjected to PCR to amplify the E2F1 promotor binding sites. The amplified fragments were then analyzed on an agarose gel. Chromatin (1%) prior to immunoprecipitation was used as the input control. The primer sequences of binding site between E2F1 and SNHG1 was as follows: SNHG1-F: 5′-CAGGAGAATTGCTTGAACCCG-3′; SNHG1-R: 5′-TGGCCCGATCTCAGCTCACT-3′.

### Nucleic acid electrophoresis

The DNA PCR products were investigated using 1% agarose gel electrophoresis with TAE running buffer. DNA was separated by electrophoresis at 100 V for 30 min. The DNA marker was Marker L (50–500 bp) (Sango Biotech, China). The bands were examined by UV irradiation (Biorad).

### Statistical analyses

The expression of SNHG1 in cancer tissues compared with normal tissues were tested by a paired t-test. Kaplan–Meier method and log-rank test were used to evaluate the survival difference between patients with high SNHG1 expression and low SNHG1 expression. The differences in the results of the in vitro and in vivo experiments between groups were analyzed using Student’s t-test. All the experiments were performed independently in triplicate. All statistical tests were two-sided, and *P* < 0.05 indicated statistical significance. Statistical analysis was performed using 332R.3.4 graphics software and GraphPad Prism software (GraphPad Software, USA).

## Supplementary Information

**Additional file 1: Figure S1.a**–**c** Higher expression level of SNHG1 was associated with poor overall survival, disease specific survival and progression free interval in UCEC. **d**–**f** Higher expression level of SNHG1 was associated with poor disease specific survival, progression free interval and disease-free interval in LIHC. **g**–**i** Higher expression level of SNHG1 was associated with poor overall survival, disease free interval and progression free interval in PRAD. **j**–**k** Higher expression level of SNHG1 was associated with poor overall survival and progression free interval in ACC. **l**–**o** Higher expression of SNHG1 was correlated with poor OS in LIHC, KIRC, SARC and UCEC.

**Additional file 2: Figure S2.** CCK-8 (**a**), wound healing (**b**) and colony formation assays (**c**) were performed to identify that silencing of TERT inhibited tumor cell proliferation and colony formation and suppressed tumor cell migration and invasion in MDA-MB-468 and Hs578T.

**Additional file 3: Table S1.** The clinical pathology information of the breast cancer tissues in the TCGA analysis for SNHG1 expression level.

**Additional file 4: Table S2.** SNHG1 expression and prognosis of human pan-cancer in TCGA database.

**Additional file 5: Table S3.** Regarding the primary samples (n = 5) validating the SNHG1 and TERT expression, patient demographic data were provided.

**Additional file 6: Table S4.** The relationship between expression of SNHG1 and TERT of human pan-cancer in TCGA database.

**Additional file 7: Table S5.** The expression profile of coding gene in breast cancer was extracted from TCGA BRCA expression profile.

**Additional file 8: Table S6**. TargetScan, and starBase databases to predict the possible miRNAs that could interact with both SNHG1 and TERT, simultaneously.

**Additional file 9: Table S7.** PROMO database was used to predict potential transcription factors (TFs) that could bind to the SNHG1 promoter.

**Additional file 10: Table S8.** The relationship between expression of E2F1 and SNHG1 of human pan-cancer in TCGA database.

**Additional file 11: Table S9.** JASPAR database was used to predict the potential binding site between E2F1 and SNHG1 promotor.

## Data Availability

All remaining data are availability within the article and Additional files, or available from the authors upon request.

## Abbreviations

ACC: Adrenocortical carcinoma
BLCA: Bladder urothelial carcinoma
BRCA: Breast carcinoma
CCK-8: Cell counting Kit-8
ceRNA: Competing endogenous RNA
CESC: Cervical and endocervical cancers
ChIP: Chromatin immunoprecipitation
CHOL: Cholangiocarcinoma
COAD: Colon adenocarcinoma
DEG: Differentially expressed gene
DSS: Disease specific survival
EMT: Epithelial mesenchymal transformation
ESCA: Esophageal carcinoma
HNSC: Head and neck squamous cell carcinoma
GEPIA: Gene Expression Profiling Interactive Analysis
KICH: Kidney chromophobe
KIRC: Kidney renal clear cell carcinoma
KIRP: Kidney renal papillary cell carcinoma
LIHC: Liver hepatocellular carcinoma
LncRNA: Long noncoding RNAs
LUAD: Lung adenocarcinoma
LUSC: Lung squamous cell carcinoma
miRNA: MicroRNA
ORF: Open reading frame
OS: Overall survival
PCPG: Pheochromocytoma and paraganglioma
PRAD: Prostate adenocarcinoma
READ: Rectum adenocarcinoma
RFS: Relapse free survival
SARC: Sarcoma
siRNA: Short interfering RNA
SNHG1: Small nucleolar RNA host gene1
STAD: Stomach adenocarcinoma
TCGA: The Cancer Genome Atlas
TERC: Telomerase RNA component
TERT: Telomerase reverse transcriptase
TF: Transcription factor
THCA: Thyroid carcinoma
TNBC: Triple negative breast cancer
UCEC: Uterine corpus endometrial carcinoma
UTRs: Untranslated regions
